# Computed Tomography Angiography and B-Mode Ultrasonography under Artificial Intelligence Plaque Segmentation Algorithm in the Perforator Localization for Preparation of Free Anterolateral Femoral Flap

**DOI:** 10.1155/2022/4764177

**Published:** 2022-09-28

**Authors:** Dan Shen, Xuehui Huang, Yinwei Huang, Dandan Zhou, Shasha Ye

**Affiliations:** Department of Hand Foot and Micro-Surgery, Yuyao People's Hospital, Ningbo 315400, Zhejiang, China

## Abstract

This research was aimed to investigate the accuracy of U-shaped network (UNet)-based computed tomography angiography (CTA) and B-mode ultrasonography (US) in the perforator localization of free anterolateral thigh flap (ALTF). Based on UNet, a fusion of deep supervision mechanism, squeeze-and-excitation module, and attention mechanism was introduced to optimize the algorithm. Then, a CTA segmentation model, DA-UNet, was established. The segmentation performance of DA-UNet and other algorithms was compared under the same conditions. 30 patients who were planned to receive ALTF surgery were selected as the research objects. According to different preoperative localization methods, they were divided into group A (CTA) and group B (B-mode US), 15 cases in each group. Combined with the actual situation during surgery, the diagnostic accordance rate, sensitivity (Sen), specificity, and the distance between the perforator location and the actual location were compared between the two groups. The Dice coefficient, Jaccard index, Sen, the area under curve (AUC), and average Hausdorff distance (AVD) of the DA-UNet segmentation algorithm were 80.70%, 69.97%, 77.56%, 0.887, and 2.48, respectively. These results were significantly better than those of other algorithms (*P* < 0.05). In group A, the diagnostic accordance rate, Sen, and specificity of patients were 96.55%, 90.52%, and 73.58%, respectively, which were higher than 91.53%, 81.36%, and 15.60% of patients in group B significantly (*P* < 0.05). There was no statistical difference in the distance between the perforator location and the actual location (*P* > 0.05). It showed that the accuracy of CTA under the UNet-based DA-UNet segmentation model in the perforator localization of ALTF was better than that of B-mode US. Thus, a reference could be provided for the preparation of free ALTF and its clinical application.

## 1. Introduction

Anterolateral thigh flap (ALTF) is a common flap transplantation technique in clinical repair and reconstruction surgery. It has the characteristics of concealed donor site, moderate skin thickness, large incision area, and the ability to be prepared into various types of flaps [1]. It is used in the preparation of fascial flaps, musculocutaneous flaps, and island flaps [2]. The ALTF feeding artery comes from the musculocutaneous perforators or septal perforators of the lateral femoral circumflex artery system. The source, course, and location of these perforators are significantly different, which increases the difficulty of flap cutting [3]. The preoperative perforator localization technique can help to better understand the anatomical structure of the perforator and its surrounding tissues, reducing the incidence of complications [4]. Preoperative perforator localization techniques mainly include computed tomography angiography (CTA), B-mode ultrasonography (US), and magnetic resonance angiography (MRA). B-mode US has the advantages of noninvasiveness, simple operation, and no site restrictions. However, B-mode US often produces false positive results, and there are defects in judging the specific location of the superficial point of deep fascia [5]. MRA has the advantages of good tissue resolution and optimal imaging selection, but its detection accuracy is poor and the diagnostic cost is high [6]. CTA has the advantages of fast scanning speed, high resolution, and noninvasiveness. Thus, it can detect the condition of the patients' flap directly and can clarify the vascular pedicle diameter and length, muscle orientation, and other related anatomical structures during the detection process [7]. However, CTA has the following shortcomings in the process of preoperative perforator localization. First, in the superficial fascia of the thigh, the development space for CTA imaging is limited, and it is difficult to grasp the time when the contrast agent reaches the peripheral blood vessels. These result in perforating vessels in the superficial fascia cannot be clearly displayed, which is easy to be missed and difficult to locate. Secondly, the preoperative localization of CTA is performed on the simulated image, so there is a certain deviation from the direct localization on the skin. Finally, it is difficult of CTA to locate the preoperative perforator by establishing a coordinate system for the anterolateral thigh area whose contour is in a curved structure. The curved structure is easy to rotate, and the deep tissue and surface skin are prone to relative displacement [8].

Traditional CTA image segmentation methods consist of region growing algorithm, active contour model, and level set method. All these methods have the shortcomings of strong artificial dependence and poor robustness in CTA image segmentation [9]. With the continuous development of artificial intelligence learning algorithms in recent years, deep learning algorithms have been widely applied in computer vision and pattern recognition. They are widely used in medical image segmentation, lesion identification, and image generation and amplification due to automatic image feature selection, powerful feature representation capabilities, and so on [10]. The fully convolutional neural network image segmentation algorithm, U-shaped network (UNet), utilizes convolution to extract features in medical image processing, so as to achieve the goal of sharing parameters. It reduces the complexity of the network model and the number of weights, but it still needs to be further optimized for its shortcomings of low segmentation rate, unsophisticated segmentation results, and poor contrast [11].

To sum up, whether the perforator can be correctly located and selected is the key to the preparation of free ALTF, while B-mode US and CTA commonly used in clinical practice have certain defects in ALTF localization. As the UNet algorithm was optimized and applied to CTA image segmentation, the application value of CTA and B-mode US image segmentation under U-net algorithm was discussed in ALTF localization. It was to provide a certain reference for the preparation of free ALTF and its clinical application.

## 2. Materials and Methods

### 2.1. UNet-Based CTA Image Segmentation Method

The network structure of UNet was mainly composed of an encoder and a decoder as shown in Figure 1. The encoder consisted of 4 downsampling layers. The input image was continuously convoluted twice and pooled to extract the global features of the image. The decoder consisted of 4 upsampling layers. After upsampling and channel merging operations on the image, the final segmentation image was output.

The resolution of the initial CTA images was relatively large, and these images could not be directly input into the UNet for training due to the limited memory of the graphics card device. The CTA images needed to be preprocessed. The coarse-to-fine (C2F) method [12] was adopted to segment the arteries in CTA images. After the upsampling of the original CTA image *I* in the coarse segmentation, the obtained coarse segmentation output image is expressed as equation (1):

(1) $$\begin{array}{c} I_{c}=U\left\{C_{s}\left[D\left(I\right)\right]\right\}. \end{array}$$

In the equation, *D* is the downsampling operation, *U* is the upsampling operation, and *C*_*s*_ is the coarse segmentation network.

In the process of fine segmentation, the CTA image was cropped and zero-padding was made in the surroundings according to *I*_*c*_ to obtain the segmentation result of the arterial cavity on the CTA image. The calculation method can be expressed as equation (2):

(2) $$\begin{array}{c} I_{o}=P\left\{F_{s}\left[C\left(I_{c},I\right)\right]\right\}. \end{array}$$

In equation (2), *P* is the zero-padding operation, *C* is the minimum circumscribed rectangle cropping operation, and *F*_*s*_ is the fine segmentation network.

### 2.2. Construction of the Optimized Algorithm under UNet

UNet had the shortcomings of unsophisticated segmentation outcomes in CTA image processing [13]. On the grounds of UNet algorithm, deep supervision mechanism, squeeze-and-excitation module, and the attention mechanism were fused and introduced for the optimization. Then, the optimized model was constructed, which was denoted as deeply supervised attention-enabled UNet (DA-UNet). For the CTA image with a resolution of *l* × *w* × *h*, the interpolation algorithm was utilized for sampling the sequence slices, so as to get the candidate segmentation results. Then, the fusion model was applied to fuse the candidate segmentation results, and the final segmentation results can be expressed as equation (3):

(3) $$\begin{array}{c} \tilde{S_{e}}=\sum_{n=1}^{N}W_{n,k}\cdot c_{n,k}+\alpha_{k},\;\left(0<k\leq A\right). \end{array}$$

Here, *A* represents the number of segmentation categories, *N* denotes the number of candidate segmentation results, and *c*_*n*,*k*_ ∈ *ℝ*^*l*×*w*×*h*^ denotes the segmentation result of the *k*-th category in the *n*-th candidate segmentation result. *W*_*n*,*k*_ ∈ *ℝ*^*l*×*w*×*h*^ represents the weighting matrix for *c*_*n*,*k*_, and *α*_*k*_ is the bias term.

Squeeze-and-excitation module could improve the expressiveness of the network through convolutional features [14]. In this work, the squeeze-and-excitation module was introduced into the UNet to weight the feature channels. After the feature map processed by convolution operation was subjected to the global average pooling operation, the spatial compression vector of the image is represented as equation (4):

(4) $$\begin{array}{c} b_{k}=\frac{1}{w\times h}\sum_{i}^{w}\sum_{j}^{h}d_{k}\left(i,j\right),\;\left(0<k\leq e\right). \end{array}$$

In equation (4), *d*_*k*_ represents the *k*-th feature channel of the feature map *D*, *D* ∈ *ℝ*^*w*×*h*×*e*^, and *e* is the number of feature map channels.

If a channel was stimulated by full connection operation twice, the descriptor $\tilde{B}$ of the channel was obtained, and its calculation method is expressed as equation (5):

(5) $$\begin{array}{c} \tilde{B}=\beta \left[w_{2}\delta \left(w_{1}B\right)\right]. \end{array}$$

In the equation above, *w*_1_ is the weight of the first full connection operation, *δ* represents the ReLU activation function, *w*_2_ is the weight of the second full connection operation, and *β* refers to the sigmoid activation function.

By weighting the feature map *D* as a weight, the output feature map $\hat{D}$ of the squeeze-and-excitation module could be obtained. The calculation method is expressed as equation (6):

(6) $$\begin{array}{c} \hat{D}=\left[{\tilde{B}}_{1}\eta_{1},{\tilde{B}}_{2}\eta_{2},\cdots ,{\tilde{B}}_{c}\eta_{c}\right]. \end{array}$$

Here, ${\tilde{B}}_{c}$ stands for the weighting of the *c*-th feature channel in the feature map *D*.

The attention mechanism was mainly in the weighted processing of the feature map [15]. As the attention mechanism was introduced into the connection layer of UNet, the shallow features of the encoder were weighted in the layer. Thereby, the optimized network paid more attention to the arterial region. For feature maps *y* and *g*, convolution layer operation and attention control processing were made after matrix addition, and the output feature map can be expressed as equation (7):

(7) $$\begin{array}{c} \hat{y}=\kappa \cdot y,\;\kappa =\beta \left[W⊗\delta \left(g+y\right)\right]. \end{array}$$

Here, W is the convolution kernel, ⊕ represents the convolution operation, *κ* refers to the attention coefficient matrix, *κ* ∈ *ℝ*^*w*×*h*^, and *g* is the feature map after upsampling as *g* ∈ *ℝ*^*w*×*h*×*e*^.

Deep supervision mechanism reduced the coarseness of image segmentation results [16]. For images of different resolutions processed by the convolution layer, the upsampling was performed, and the output image was obtained after normalization by Softmax. It is calculated using equation (8):

(8) $$\begin{array}{c} O_{u}=\text{softmax}\left\{fs_{1}+U\left[fs_{2}+U\left(fs_{3}+U\left(fs_{4}\right)\right)\right]\right\}. \end{array}$$

In the equation, *f*_*s*_ represents different resolutions, and *U* is the upsampling operation.

The output image processed by the DA-UNet contained the probability value of each pixel classified as background or carotid artery in the input image. A loss function was needed to evaluate the difference between the segmentation result and the gold standard. In this work, the classification cross entropy loss (CEL) was used for the evaluation of the mechanical energy of DA-UNet processing. CEL is expressed as equation (9):

(9) $$\begin{array}{c} C\left(Z,z\right)=-\frac{1}{M}\sum_{m=1}^{M}\sum_{k=1}^{e}Z_{m}\log\;Z_{m}^{k}. \end{array}$$

Here, *M* is the number of pixels in a batch of images in the training, and *e* is the number of pixel categories. *Z*_*m*_^*k*^ represents the binary label of pixel *m* for category *k* in the gold standard *Z*, while *z*_*m*_^*k*^ represents the probability that pixel *n* belongs to the category *k* in the segmentation result *z*.

Figure 2 displays the CTA image processing flow of the DA-UNet algorithm under the UNet. First, the initial number of convolution kernels in the network was set, and the convolution operation was performed on the input CTA image. The batch normalization and maximum pooling operations were added to the image blocks, and then the layer-by-layer downsampling operation was made for Max pooling. The downsampled image was subjected to upsampling operation in the decoder, convolution channel weighting processing, connection layer mechanism module, attention mechanism processing, and finally the output layer deep supervision mechanism. Afterwards, the output of each upsampling layer was superimposed with the final output, a segmented CTA image was obtained.

### 2.3. Evaluation Indicators of CTA Image Segmentation

The CTA image segmentation was evaluated using Dice coefficient, Jaccard index, sensitivity (Sen), area under the receiver operator characteristic curve (AUC), and average Hausdorff distance (AVD) in this work. The Dice coefficient mainly evaluated the overlapping rate between the segmentation result region and the gold standard region, with the range of [0, 1]. The Dice coefficient is calculated using equation (10):

(10) $$\begin{array}{c} \text{Dice}\left(A,B\right)=\frac{2\left|A\cap B\right|}{\left|A\right|+\left|B\right|}=\frac{2\text{TP}}{2\text{TP}+\text{FP}+\text{FN}}. \end{array}$$

The Jaccard index was a measure of regional overlapping [17], which is calculated using equation (11):

(11) $$\begin{array}{c} \text{Jaccard}=\frac{\left|A\cap B\right|}{\left|A\cup B\right|}=\frac{\text{TP}}{\text{TP}+\text{FP}+\text{FN}}. \end{array}$$

Sensitivity (Sen) was utilized to measure the probability that a voxel that was positive in the gold standard was also positive in the segmentation result, and it is calculated using equation (12):

(12) $$\begin{array}{c} \text{Sen}=\frac{\text{TP}}{\text{TP}+\text{FN}}. \end{array}$$

AUC was used to measure the classification accuracy of voxels in the segmentation results, and its calculation method is expressed as equation (13):

(13) $$\begin{array}{c} \text{AUC}=1-\frac{1}{2}\left(\frac{\text{FP}}{\text{FP}+\text{TN}}+\frac{\text{FN}}{\text{FN}+\text{TP}}\right). \end{array}$$

AVD was an evaluation method for image segmentation under spatial distance, and its calculation is described as equation (14):

(14) $$\begin{array}{c} \text{AVD}\left(A,B\right)=\frac{\left|B\right|-\left|A\right|}{\left|A\right|}. \end{array}$$

In equations (10)–(14), TP, FN, TN, and FP represent the number of true positives, false negatives, true negatives, and false positives, respectively. *A* is the model segmentation result, while *B* is the gold standard.

For the experimental environment, the model of central processing unit was Intel(R) Core(TM) i7-7800X, with the main frequency of 3.50 GHz, the memory of 16 *G*, the operating system of Linux, and the programming language of Python 3.6.6. The Dice coefficient, Jaccard index, Sen, AUC, and AVD of UNet, DA-UNet, 3D-UNet [18], Isensee-UNet [19], and RA-UNet [20] algorithms were compared under the same conditions.

### 2.4. Research Objects and Groups

Thirty patients admitted to the hospital from June 2018 to June 2020, who were to undergo ALTF surgery, were included as the research objects. These patients were randomly divided into group A (15 cases) and group B (15 cases). In group A, CTA was used for the perforator localization of the free ALTF; in group B, the simple perforator localization of the free ALTF was given. The age range of the included objects was 18–60 years old, with an average age of (34.62 ± 6.75) years old; 23 males and 7 females were included. The experimental process had been approved by the ethics committee of the hospital, and all objects included signed the informed consent forms.

Inclusion criteria were as follows: (1) patients were between the ages of 18 and 60 years old, regardless of gender; and (2) patients had skin and soft tissue defects of the limbs. The exclusion criteria were as follows: (1) patients had a history of iodine allergy; (2) patients had the positive result of iodine allergy test; (3) patients' lateral circumflex femoral artery was determined as the type without thick branches; (4) patients suffered from liver or kidney dysfunction (glutamic-pyruvic transaminase >80 U/L); (5) patients got pulmonary infection shown in chest X-ray examination; (6) patients had renal insufficiency (creatinine >200 mg/L); (7) patients had a cardiac function > grade II; (8) local ulcers in patients were diagnosed as malignant tumors; (9) patients had a history of mental illness once; (11) patients got severe allergic reactions during CTA examination; (12) patients had an anesthesia accident during anesthesia, which made the surgery could not be performed; and (13) the lateral femoral circumflex artery was classified with no thick branch during the surgery, or they went with poor vascular conditions.

### 2.5. B-Mode US, CTA, and Image Processing

B-mode US was performed on patients using color B-mode US diagnostic apparatus, with LA523 high-frequency probe, and the probe frequency was 8–12 MHz. For the B-mode US examination, the supine position should be taken. The midpoint of the line connecting the skeleton was taken as the point *M*, and the probe was perpendicular to the skin surface. In the two-dimensional images, the rectus femoris, vastus lateralis, vastus intermedius, vastus medialis, etc., were observed. The main, ascending, transverse, and descending branches of the femoral artery and lateral femoral circumflex artery were also observed in the blood flow images. The running region of the descending branch of the lateral femoral circumflex artery was determined. The midpoint *M* as the center of the circle, and the perforating vessel in the direction of the vastus lateralis muscle that located the descending branch of the lateral femoral circumflex artery was sought. After the perforating vessel in the direction of the vastus lateralis muscle was detected, the distance from the *M* point was measured immediately, which was marked on the body surface with gentian violet.

The patients were scanned in the supine position using the Toshiba Aquilion ViSION 320-row computed tomography scanner. The scanning range was from the anterior superior iliac spine to the lower edge of the patella. Iopromide injection was used as a contrast agent, at a dose of 370 mgI/mL and an injection rate of 5 m/s. The scanning parameters included the voltage 120 KV, current 300 mA, field of view 250–400 mm, slice thickness 0.5 mm for reconstruction, and reconstruction slice spacing 0.3 mm. For the scanning method, after iopromide injection was injected through the cubital vein with a high-pressure syringe, the automatic monitoring and trigger scanning mode was adopted. The layer of the bifurcation of the main femoral artery was taken as the monitoring layer, and the region of interest (ROI) was set at the layer of the femoral artery. When the CTA value in the ROI reached 280 HU, the arterial phase scanning was automatically triggered.

After the scanning was completed, the CTA volume data of patients were imported into the three-dimensional image workstation for processing. Multiplanar reconstruction, maximum intensity projection, curved planar reconstruction, vessel probe, volume reconstruction (VR), and other three-dimensional postprocessing techniques were utilized for observation of the lateral femoral artery and its branches. In the CTA images, the morphology of the lateral circumflex femoral descending artery and the location of the perforator were observed. The location of the perforator was located in VR mode according to the points of interest. Meanwhile, the iliac-patellar line was drawn, connecting the anterior superior iliac spine to the lateral border of the patella. The midpoint of the line was taken as the center, and then a three-dimensional coordinate system was constructed. Its spatial position was accurately measured through the projection point of the perforator on its surface skin.

### 2.6. Surgical Methods and Postoperative Treatment

Referring to the method of Tsai [21], free flap transplantation was performed and improved. All patients were given systemic support before surgery to correct their anemia, hypoalbuminemia, and electrolyte imbalance. Debridement and vacuum sealing drainage were performed in the recipient area, and the surgery was performed after the infection was significantly controlled. The surgery was performed in a supine position, and continuous epidural spinal anesthesia combined with block anesthesia or general anesthesia was used. After routine disinfection and surgical draping, the chief surgeon marked the perforation point with reference to the preoperative B-mode US or CTA measurement. With the shape and area of the wound in the recipient area, the patient's skin flap implantation was designed to remove the free skin flap. The upper, lower, and outer edges of the patient's skin flap were incised, and the deep fascia and subcutaneous tissue were fixed and sutured. The flap was lifted slowly, and the subcutaneous perforating artery was found. Then, the actual position on the body surface of the perforator was compared with the results of CTA and B-mode US examinations. The length of the perforator was measured with a sterilized stainless ruler, and the relevant information was recorded. The vascular pedicle was freed to the root of the perforator by the join-forces traction method, and the flap was completely incised along the periphery of the flap. The flap was lifted from the deep surface and then was removed; the vascular bundle arteries and veins were trimmed under the microscope, and the vascular pedicle was connected with the blood supplying arteries and veins of the recipient area. After anastomosis, the vascular clip was loosened, and the arterial pulsation and venous filling were observed. The wound was closed, the drainage fluid was drained, and then the wound was bandaged. The wound in the donor area of the thigh was roped in and sutured. For the wound that cannot be eliminated, epidermis or autologous medium-thickness skin grafts on the head, abdomen, etc., were taken for repair and transplantation.

The patients were treated with routine anticoagulation, anti-infection, antispasmodic, and baking lamp irradiation after surgery. The drainage tube was removed 3–4 days after receiving subcutaneous drainage. The color, temperature, and filling time of capillaries of the transplanted skin ALTF were closely monitored after surgery. If the patient had a vascular crisis, it should be treated in time.

### 2.7. Statistical Methods

The experimental data were processed with SPSS19.0. The distance between the location of perforator on the branch surface and the perforator location confirmed during the surgery was expressed as the mean ± standard deviation ($\bar{x}\pm s$). The measurement data between the two groups were compared by the *t* test. The enumeration data were expressed as percentage (%) and was tested using the *χ*^*2*^ test. *P* < 0.05 indicated that the difference was statistically significant.

## 3. Results and Analysis

### 3.1. Comparison of Dice Coefficient of Femoral Artery in CTA Images Segmented by Different Algorithms

The Dice values of UNet, DA-UNet, 3D-UNet, Isensee-UNet, and RA-UNet algorithms were compared under the same circumstances, which are shown in Figure 3. The Dice coefficient of UNet, DA-UNet, 3D-UNet, Isensee-UNet, and RA-UNet were 64.05%, 91.87%, 75.92%, 70.19%, and 67.54%, respectively. The Dice value of DA-UNet was remarkably higher than that of other algorithms (*P* < 0.05).

### 3.2. Comparison of Jaccard Index and Sen of Femoral Artery in CTA Images Segmented by Different Algorithms

The comparison of Jaccard index and Sen of different algorithms is presented in Figure 4. The Jaccard index and Sen of the DA-UNet algorithm were 85.22% and 90.03%, respectively, markedly higher than those of other algorithms (*P* < 0.05).

### 3.3. Comparison of AUC and AVD of Femoral Artery in CTA Images under Different Algorithms

The comparison of AUC and AVD of different algorithms is presented in Figure 5. The AUC of the DA-UNet algorithm was 0.933, and the AVD of DA-UNet was 0.19. The AUC of the DA-UNet algorithm was higher than that of other algorithms (*P* < 0.05), but its AVD value was observably lower than that of other algorithms (*P* < 0.01).

### 3.4. Comparison of Basic Data of Patients between the Two Groups

The age, gender ratio, and skin defect range of the two groups of patients were compared. There was no significant difference in age, gender ratio, as well as skin defect range between group A and group B (*P* > 0.05), which can be seen in Table 1.

### 3.5. Comparison of the Causes of Injury and Injured Sites

The causes of injury and injured sites of patients in the two groups were compared and analyzed, as shown in Figures 6 and 7. In group A, 2 cases (13.33%), 3 cases (20.00%), 1 case (6.67%), 1 case (6.67%), 2 cases (13.33%), 3 cases (20.00%), and 3 cases (20.00%) were injured by heavy objects, traffic accidents, mechanical crushing, falling from a height, ulcers, postoperation, and infections, respectively. In group B, 3 cases (20.00%), 2 cases (13.33%), 1 case (6.67%), 1 case (6.67%), 3 cases (20.00%), 3 cases (20.00%), and 2 cases (13.33%) were injured by heavy objects, traffic accidents, mechanical crushing, falling from a height, ulcers, postoperation, and infections, respectively. No significant difference was found in the proportion of patients with different causes of injury and injured sites between group A and group B (*P* > 0.05).

### 3.6. Analysis of Preoperative Localization Characteristics

The distance between the preoperative perforator position and the actual position determined during surgery was compared between groups, which is shown in Figure 8. Under CTA, the distance between the preoperative perforator position on body surface and the actual position in group A was (11.26 ± 4.76) mm, and that under B-mode US in group B was (12.45 ± 5.12) mm. There was no significant difference between the two groups in the distance between the perforator position and the actual position (*P* > 0.05).

The diagnostic accordance rate, Sen, and specificity of patients in group A and group B are compared in Figure 9. The number of perforators found during surgery in group A and group B was 58 and 59, respectively. The diagnostic accordance rate, Sen, and specificity of patients in group A were 96.55%, 90.52%, and 73.58%, respectively; those in group B were 91.53%, 81.36%, and 15.60%, respectively. The diagnostic accordance rate, Sen, and specificity of group A patients were all significantly higher than those in group B (*P* < 0.01).

## 4. Discussion

CTA is used for the clinical body surface localization of perforating vessels because of its high image resolution. This method can shorten the operation time of patients, reduce the incidence of postoperative complications, and reduce the postoperative burden of patients [22]. CTA has significant advantages in the diagnosis of vascular lesions, visualization of blood vessels, and quantitative analysis of anatomical information, which made CTA become the gold standard for preoperative design of breast reconstruction [23]. However, there are still some deviations in the examination process. With the shortcomings of CTA images, UNet was optimized and applied to the segmentation of arterial blood vessels in CTA images in this research. The results demonstrated that the Dice coefficient, Jaccard index, Sen, AUC, and AVD of DA-UNet were greatly better than those of other algorithms (*P* < 0.05). It was suggested that the performance of the UNet-based DA-UNet algorithm in femoral artery segmentation of CTA images was highly improved perhaps because the C2F segmentation method was adopted. Moreover, the deep supervision mechanism, squeeze-and-excitation module, and attention mechanism were fused and introduced in the optimization. The combination of these optimization methods made the DA-UNet algorithm significantly improve the accuracy of CTA image segmentation, while reducing the loss of resolution. Elgohary et al. [24] established the C2F-3D-UNet under UNet algorithm and applied it to CTA image segmentation. The results indicated that the Dice value, Jaccard index, Sen, AUC, and AVD for CTA image segmentation were 80.70%, 69.97%, 77.56%, 0.887, and 2.48, respectively. The corresponding values in the results of this work were notably higher than those of the network, suggesting that the DA-UNet in this work had a potential application value in CTA image segmentation.

The results of this work found no significant difference in the distance between the perforator position and the actual position of patients between group A and group B (*P* > 0.05). The diagnostic accordance rate, Sen, and specificity of patients in group A were remarkably higher than those in group B (*P* < 0.01). The accuracy, Sen, and specificity of CTA were higher than those of B-mode US. However, there was still a certain deviation between the perforator location examined by CTA and the actual location. This might be because the images obtained from CTA examination were three-dimensional postprocessing images, and the image processing led to some difference between the location and the actual location [25]. On the other hand, it might be related to factors such as the body position in CTA examination and that during the surgery, which resulted in the rotation of the lower extremity. During the surgery, the traction of tension was combined after the fascia and skin were incised, so the position of the out point of perforator changed [26]. Therefore, it was necessary to simulate the intraoperative body position performance in the clinical practice, so as to improve the accuracy of CTA examination. In conclusion, CTA under the UNet algorithm had a definite advantage over B-mode US in perforator localization of ALTF, which was similar to the findings of Ma et al. [27].

## 5. Conclusion

The accuracy of UNet-based CTA and B-mode US were analyzed in the perforator localization in the preparation of free ALTF. The accuracy of CTA under UNet was better than that of B-mode US in the perforator localization of ALTF. However, there were still some deficiencies in this research. The number of patients included was limited, the follow-up time was short, and the incidence of postoperative adverse events in patients was not analyzed in detail. In the future work, the sample size would be expanded, and the incidence of adverse events would be counted to further clarify the mid-term and long-term clinical effects of these two methods. All in all, this work provided a reference for the preparation of free ALTF and its clinical application.

## Figures and Tables

**Figure 1:** Image processing flow of UNet.

**Figure 2:** Flow chart of CTA image processing by DA-UNet algorithm.

**Figure 3:** Comparison of Dice coefficients of CTA images segmented by different algorithms. ^*∗*^Compared with DA-UNet algorithm, *P* < 0.05.

**Figure 4:** Comparison of Jaccard index and Sen of CTA images segmentation by different algorithms. ^*∗*^Compared with those of DA-UNet algorithm, *P* < 0.05.

**Figure 5:** Comparison of AUC and AVD values of different algorithms. ^*∗*^Compared with other algorithms, *P* < 0.05; while ^*∗∗*^compared with other algorithms, *P* < 0.01.

**Figure 6:** Comparison of the causes of injury between the two groups.

**Figure 7:** Comparison of injured sites of patients between the two groups.

**Figure 8:** Comparison of the distance between the preoperative perforator position and the actual position in two groups.

**Figure 9:** Comparison of accordance rate, Sen, and specificity for preoperative localization in different groups. ^*∗∗*^Compared with group B, *P* < 0.01.

**Table 1:** Comparison of basic data of the two groups.

Groups	Group A (*n* = 15)	Group B (*n* = 15)	*t* or *χ*^*2*^	*P* value

Age (years old)	34.15 ± 9.27	35.27 ± 10.42	2.224	0.325
Male [cases, (%)]	11 (73.33)	12 (80.00)	2.458	0.283
Female [cases, (%)]	4 (26.67)	3 (20.00)		
Skin defect range (cm)	8.70 × 12.83–28.40 × 24.16	8.51 × 12.24–29.14 × 25.23	3.025	0.146

## Data Availability

The data used to support the findings of this study are available from the corresponding author upon request.
